The article "RNA interference-mediated USP22 gene silencing promotes human brain glioma apoptosis and induces cell cycle arrest" was retracted in 2023. Reasons: duplicated images; signs of a paper mill.

# RNA interference-mediated USP22 gene silencing promotes human brain glioma apoptosis and induces cell cycle arrest

**DOI:** 10.3892/ol.2013.1188

**Published:** 2013-02-12

**Authors:** ZHAO HUI LI, YIN YU, CHAO DU, HONG FU, JIAN WANG, YU TIAN

**Affiliations:** 1 Department of Neurosurgery, China-Japan Union Hospital of Jilin University, Changchun 130033;; 2 Department of Neurosurgery, Affiliated Hospital of Inner Mongolia University for Nationalities, Tongliao 028000, P.R. China

**Keywords:** RNA interference, USP22 gene, human brain glioma, cell apoptosis, cell cycle

## Abstract

Ubiquitin-specific protease 22 (USP22) is a novel tumor stem cell marker that plays a key role in tumorigenesis and cell cycle progression. However, the effect of silencing the USP22 gene on human brain glioma cell growth is not well understood. In the present study, high gene expression of USP22 was identified in human brain glioma cells. In addition, RNA interference technology was used to silence USP22 gene expression in human brain glioma cells. Silencing the USP22 gene was found to effectively inhibit proliferation of human brain glioma cells, resulting in cell apoptosis and cell cycle arrest at the G_2_/M phase. USP22 silencing was also found to lead to reduced expression of cell cycle proteins, including CDK1, CDK2 and CyclinB1. In summary, in this study the USP22 gene was demonstrated to play a key regulatory role in the growth of human brain glioma cells by affecting progression of apoptosis and the cell cycle.

## Introduction

Originating in the nerve epithelial tissue, brain glioma is one of the most common malignant tumors in the central nervous system accounting for >70% of primary malignant brain tumors (1–3). The high incidence, poor prognosis and low efficacy of therapeutics associated with brain glioma has attracted considerable attention from researchers in the central nervous system disease field; however, progress remains challenging (4). At present, brain glioma is largely treated with surgery, radiotherapy and chemotherapy; however, the curative effect and prognosis are far from optimistic, and there is no significant improvement in treatment efficacy of brain glioma (5–7). In addition, current knowledge on the molecular mechanism of the generation and development of brain glioma remains extremely limited. Analysis of the roles played by specific molecules in the brain glioma generation and development process is important for the identification of effective treatment approaches and may provide effective molecular targets for future molecular therapies.

A previous study identified an 11-gene Polycomb/cancer stem cell signature that may predict the probability of treatment failure in cancer patients (8). Ubiquitin-specific protease 22 (USP22) is a novel putative cancer stem cell marker involved in the 11-gene Polycomb/cancer stem cell signature (9). USP22 belongs to a large family of proteins with ubiquitin hydrolase activity and has been identified to be an important subunit of the human Spt-Ada-Gcn5 acetyltransferase (hSAGA) transcriptional cofactor complex, which is required for activator-driven transcription and cell cycle progression. Within hSAGA, USP22 removes ubiquitin from histone H2B, thus regulating the transcription of downstream genes associated with epigenetic alteration and cancer progression.

The article "RNA interference-mediated USP22 gene silencing promotes human brain glioma apoptosis and induces cell cycle arrest" was retracted in 2023. Reasons: duplicated images; signs of a paper mill.

A number of previous studies have reported high expression of USP22 in specific malignant tumors, affecting the progression and prognosis of malignant tumors, including esophageal carcinoma and gastric, colorectal and breast cancer (10–13). To date, the expression of USP22 in human brain glioma cells and its role in cell growth has not been determined. In the present study, high expression of USP22 in human brain glioma cells was identified. RNA interference was used to silence the USP22 gene, leading to apoptosis of human brain glioma cells and induction of cell cycle arrest. In addition, USP22 has been reported to be required for the correct function of MYC, which is widely hypothesized to play a significant role in the regulation of the tumor cell cycle and tumor invasion (14). USP22 has also been demonstrated to inhibit transcription of the p21 gene by deubiquitinating the transcriptional regulator, FBP1, leading to cell proliferation and tumorigenesis (15).

The aim of the present study is to determine the *in vitro* effect of USP22 gene silencing by RNA interference on human brain glioma cell apoptosis and the cell cycle and to elucidate its molecular mechanism.

## Materials and methods

### Cell culture

Human brain glioma U87 and U251 cells were purchased from American Type Culture Collection (Manassas, VA, USA). Cells were cultured in Dulbecco's modified Eagle's medium (DMEM; Gibco-BRL, Carlsbad, CA, USA) containing 10% fetal calf serum (Hyclone Laboratories, Inc., Logan, UT, USA), 100 U/ml penicillin and 100 U/ml streptomycin in an incubator containing 5% CO_2_ and 95% O_2_ at 37°C. Experimental analyses were performed when cells reached logarithmic growth phase.

The study was approved by the Ethics Committee of the China-Japan Union Hospital of Jilin University, Changchun, China.

### Small interfering RNA (siRNA) transfection

Human brain glioma cells were inoculated in 6-well culture plates containing DMEM in the absence of antibiotics at a density of 5×10^5^ cell/ml. Transfection was performed when the cells reached >60% confluence. siRNA and Lipofectamine 2000 were added according to the manufacturer's instructions, as described previously (Invitrogen, Carlsbad, CA, USA) (16). The USP22 siRNA sequence was as follows: sense 5′-CACGGACAGUCUCAACAAUTT-3′ and anti-sense 5′-AUUGUUGAGACUGUCCGUGTT-3′. Non-specific control siRNA was used as the control group. The efficiency of siRNA interference was determined by RT-PCR and western blot analysis.

The article "RNA interference-mediated USP22 gene silencing promotes human brain glioma apoptosis and induces cell cycle arrest" was retracted in 2023. Reasons: duplicated images; signs of a paper mill.

### RNA extraction and RT-PCR determination

Total RNA was extracted from each experimental group and RNA concentration was calculated according to the manufacturer's instructions (RNAisoTM Plus; Takara Bio, Inc., Shiga, Japan). RT-PCR was performed using a RT-PCR kit obtained from Takara Bio, Inc. and performed in accordance with the manufacturer's instructions. USP22 and β-actin primers were synthesized by Invitrogen Life Technologies (Carlsbad, CA, USA). The primers for amplification were as follows: USP22, 5′-GGACAACTGGAAGCAGAACC-3′ (forward) and 5′-TGAAACAGCCGAAGAAGACA-3′ (reverse); β-actin, 5′-CTGGGACGACATGGAGAAAA-3′ (forward) and 5′-AAGGAAGGCTGGAAGAGTGC-3′ (reverse). Reaction conditions were as follows: 94°C for 2 min followed by 34 cycles of degradation at 94°C for 30 sec, annealing at 61°C for 30 sec and extension at 72°C for 30 sec. PCR products were subjected to electrophoresis on a 1.0% agarose gel, then scanned and analyzed with a gel imaging system.

### Western blot analysis

Cells of all experimental groups were collected using a cell scraper and 2 ml lysis solution (50 mM Tris-HCl, 137 mM NaCl, 10% glycerin, 100 mM sodium vana-date, 1 mM PMSF, 10 mg/ml aprotinin, 10 mg/ml leupeptin, 1% NP-40 and 5 mM cocktail containing protease inhibitors; pH 7.4) was added to extract proteins. Protein concentation was determined by the BCA method rationing and separated by SDS-PAGE. Next, proteins were transferred to PVDF membranes using the semi-dry method and blocked overnight using 5% skimmed milk powder at 4°C. Membranes were washed with TBST and incubated for 1 h at 37°C with primary antibodies against target proteins, followed by an additional TBST wash. Membranes were incubated with appropriate secondary antibodies for 1 h at 37°C and washed with TBST. Antibody reactions were developed by color reaction for 5 min using autoradiography and Quantity One (Bio-Rad, Hercules, CA, USA) was used to perform optical density analysis and quantification.

### Cell viability

Cell viability was determined using the MTT method. Cells (2×10^4^ cell/well) were cultured in 96-well culture plates 1 day prior to siRNA transfection. Following adherence to the culture plates, cells were transfected with USP22 and control siRNA on day 2. MTT solution (5 mg/ml; 20 μl) was added to each well and cells were cultured in a CO_2_ incubator for 4 h. Following this, the culture solution was removed and 150 μl DMSO was added to each well and agitated at room temperature for 10 min. OD values of each well were measured using a microplate reader. Analysis for each experimental group was performed in six double wells. Average values were calculated and the growth curves were constructed.

The article "RNA interference-mediated USP22 gene silencing promotes human brain glioma apoptosis and induces cell cycle arrest" was retracted in 2023. Reasons: duplicated images; signs of a paper mill.

### Test of apoptosis with flow cytometry

Cells from all experimental groups were digested in 0.25% trypsin and resuspended in PBS to prepare single cell suspensions. Cell density was adjusted to 1×10^6^ cell/ml. Next, 5 μl Annexin V-FITC and 5 ml PI were added and cells were incubated for 30 min at 4°C prior to analysis by flow cytometry.

### Cell cycle analysis

Cells were collected using the trypsin method and washed 3 times with PBS. Following this, cells were fixed at 4°C using 75% cold ethanol overnight. Ethanol was removed and cells were washed 3 times with PBS. Cell density was adjusted to 1×10^6^ cells/ml at a final volume of 100 μl DNAStain comprehensive dye liquor (500 ml; with final concentrations of 50 mg/l RNase, 100 mg/l PI and 1 mg/l Triton X-100) for storage at room temperature in the dark for 15 min prior to analysis by flow cytometry.

### Statistical analysis

SPSS 16.0 statistical software was used for statistical analysis. Values are presented as mean ± SD. Statistical analysis was performed using the Student's t-test. P<0.05 was considered to indicate a statistically significant difference.

## Results

### USP22 gene expression in human brain glioma cells

USP22 gene expression was analyzed by RT-PCR. USP22 mRNA was highly expressed in U87 and U251 cells of human brain glioma and USP22 mRNA expression was higher in U87 cells. In addition, western blot analysis of USP22 protein expression identified that protein levels in U87 and U251 cells were consistent with those of USP22 mRNA. The results indicate that USP22 mRNA and protein are expressed at high levels in U87 and U251 cells of human brain glioma (Fig. 1).

### RNA interference-mediated USP22 gene silencing in human brain glioma cells

RNA interference was performed by transfecting U87 and U251 cells with control and USP22 siRNA. Following transfection, RT-PCR and western blot analysis were performed to determine USP22 mRNA and protein expression levels. USP22 siRNA transfection (58 nM) for 24 h was observed to significantly reduce expression of USP22 mRNA and protein in U87 and U251 cells (Fig. 2A–C). These results indicate that USP22 siRNA transfection for 24 h effectively silenced USP22 gene and protein expression.

The article "RNA interference-mediated USP22 gene silencing promotes human brain glioma apoptosis and induces cell cycle arrest" was retracted in 2023. Reasons: duplicated images; signs of a paper mill.

### RNA interference-mediated USP22 gene silencing and growth inhibition of human brain glioma cells

To investigate whether RNA interference-mediated USP22 gene silencing affects the growth of human brain glioma cells, the MTT method was used to analyze the viability of U87 and U251 cells at 12, 24, 48, 72 and 96 h following transfection with USP22 siRNA. The results indicate that the viability of U87 and U251 cells was significantly reduced compared with the control and control siRNA groups. These observations indicate that USP22 gene silencing by RNA interference inhibits growth of human brain glioma cells (Fig. 3A and B).

### RNA interference-mediated USP22 gene silencing induced apoptosis of human brain glioma cells

To investigate the molecular mechanism by which USP22 silencing inhibits human brain glioma cell growth, flow cytometry was used to determine the rate of cell apoptosis and western blot analysis was performed to analyze expression levels of apoptosis-related protein changes. Following RNA interference-mediated USP22 gene silencing (24 h), the apoptosis rate of U87 and U251 cells was found to increase significantly (Fig. 4A and B). In addition, protein expression levels of procaspase-9, -8 and -3 were markedly reduced (Fig. 4C and D). The results indicate that inhibition of human brain glioma cell growth by USP22 gene silencing may be relevant to cell apoptosis.

### USP22 gene silencing resulted in cell cycle arrest of human brain glioma cells in the G_2_/M phase

To determine the molecular mechanism by which USP22 gene silencing leads to inhibition of human brain glioma cell growth, the cell cycle was analyzed using flow cytometry. The percentage of USP22 siRNA-transfected U87 and U251 cells entering the G_2_/M phase was significantly higher than that of the control siRNA group (Fig. 5A and B), indicating that the majority of the cells were arrested in the G_2_/M phase. In addition, expression of cell cycle proteins, including CDK1, CDK2, CyclinB1 and CyclinD1, were analyzed by western blot analysis. CDK1, CDK2 and CyclinB1 expression in USP22 siRNA-transfected U87 and U251 cells was markedly reduced. By contrast, the expression of CyclinD1 protein was unchanged (Fig. 6A and B). The results indicate that inhibition of human brain glioma cell growth by USP22 gene silencing may induce G_2_/M phase cell cycle arrest via the downregulation of CDK1, CDK2 and CyclinB1 protein expression.

## Discussion

USP22 was recently identified as a novel human deubiquitinating enzyme. High expression levels of USP22 are used to predict the time of recurrence, distant metastasis and treatment failure and correlate with poor prognosis in a number of types of tumor (11,17,18). Previous studies have reported that USP22 silencing inhibits the proliferation of various tumor cells (19–21). However, little is known with regards to the effect of USP22 gene silencing in human brain glioma cells. Therefore, the present study aimed to determine the role of USP22 in human brain glioma and its molecular mechanism. RT-PCR and western blot analysis were performed, revealing high USP22 gene and protein expression in human brain glioma cells, and indicating that USP22 gene expression may represent a novel biological marker and treatment target for brain glioma.

The article "RNA interference-mediated USP22 gene silencing promotes human brain glioma apoptosis and induces cell cycle arrest" was retracted in 2023. Reasons: duplicated images; signs of a paper mill.

To establish the effect of the USP22 gene on human brain glioma, small RNA interfering technology was utilized to silence USP22 gene expression in human brain glioma cells. Following this, the biological status of the brain glioma cells was analyzed. Following USP22 gene silencing, the replication rate of brain glioma cells was markedly reduced, indicating that the USP22 gene is involved in the regulation of human brain glioma cell proliferation. Previous studies have demonstrated that the USP22 gene promotes the proliferation of esophageal carcinoma (10) and lung (22) breast (13), colorectal (21) and bladder cancer cells (20). Consistent with these observations, in the present study, USP22 was demonstrated to play an important role in the regulation of human brain glioma cell proliferation.

However, the mechanism by which USPCC gene silencing leads to inhibition of human brain glioma cell proliferation remains unknown. Flow cytometry analysis revealed that human brain glioma cell apoptosis occurred following USP22 gene silencing. Previous studies have reported that USP22 gene silencing induced apoptosis of bladder (20) and colorectal cancer cells (21). Consistent with these results, in the current study, USP22 inhibition of human brain glioma cell proliferation was hypothesized to be markedly associated with apoptosis. In addition, protein expression of procaspase-9, -8 and -3 was found to be significantly reduced following USP22 gene silencing. The activation of members of the caspase family is an important prerequisite for apoptosis (23). The rate of cell apoptosis was also found to increase, indicating that USP22 gene silencing may induce this process in brain glioma cells. Analysis by flow cytometry revealed that USP22 gene silencing arrested human brain glioma cells in the G_2_/M phase. In addition, expression of cell cycle regulatory proteins, including CDK1, CDK2 and CyclinB1, was markedly reduced while no change in the expression of CyclinD1 was identified. These observations indicate that USP22 gene silencing leads to the reduction in the number of human brain glioma undergoing cell division and subsequent inhibition of cell replication.

The article "RNA interference-mediated USP22 gene silencing promotes human brain glioma apoptosis and induces cell cycle arrest" was retracted in 2023. Reasons: duplicated images; signs of a paper mill.

In the present study, high expression of the USP22 gene in human brain glioma cells was identified for the first time and USP22 gene silencing was found to inhibit human brain glioma cell replication via induction of apoptosis and cell cycle arrest. These observations indicate that the USP22 gene may represent a novel molecular targeted approach for future treatment of brain glioma.

## Figures and Tables

**Figure 1:** USP22 gene and protein expression in human brain glioma cells. (A) USP22 mRNA expression via RT-PCR analysis. (B) USP22 protein expression via western blot analysis. (C) Histogram of USP22 gene expression levels. Each independent experiment was repeated 3 times. USP22, ubiquitin-specific protease 22.

**Figure 2:** RNA interference to silence USP22 gene expression in human brain glioma cells. U87 and U251 cells were transfected with USP22 siRNA for 24 h (A) RT-PCR and (B) western blot analysis to determine interference efficiency following transfection. USP22, ubiquitin-specific protease 22.

**Figure 3:** USP22 gene silencing inhibits human brain glioma cell growth. MTT was performed to analyze viability of (A) U87 and (B) U251 cells following transfection with USP22 siRNA. Each independent experiment was repeated 3 times. USP22, ubiquitin-specific protease 22.

**Figure 4:** USP22 gene silencing led to human brain glioma cell apoptosis. (A) Flow cytometry to analyze cell apoptosis rate. (B) Quantification of cell apoptosis rate (%) in U87 and U251 cells. (C) Western blot analysis of procaspase-9, -8 and -3 protein expression. (D) Quantification of procaspase-9, -8 and -3 protein expression (%). Each independent experiment was performed 3 times. P<0.05, vs. control. USP22, ubiquitin-specific protease 22.

**Figure 5:** USP22 gene silencing arrested human brain glioma cells in the G_2_/M phase. (A) Flow cytometry to analyze cycle changes in U87 and U251 cells. (B) Quantification of cell cycle changes (%). Each independent experiment was performed 3 times.^*^P<0.05, vs. control. USP22, ubiquitin-specific protease 22.

**Figure 6:** USP22 gene silencing downregulated the expression of CDK1, CDK2 and CyclinB1 protein. (A) Western blot analysis of protein expression of CDK1, CDK2, CyclinB1 and CyclinD1 proteins. (B) Quantification of protein expression of CDK1, CDK2, CyclinB1 and CyclinD1 (%). ^*^P<0.05, vs. control. Each independent experiment was performed 3 times. USP22, ubiquitin-specific protease 22.
